# Design and Performance Analysis of a Mecanum-Built Perturbation-Based Balance Training Device

**DOI:** 10.1155/2024/3622556

**Published:** 2024-03-29

**Authors:** Jaison Jacob Mathunny, Hari Krishnan S, Ashokkumar Devaraj, Varshini Karthik

**Affiliations:** Department of Biomedical Engineering, SRM Institute of Science and Technology, Kattankulathur 603203, Tamil Nadu, India

## Abstract

This study proposes a mecanum-built perturbation-based balance training device aimed at improving motor adaptive skills for fall prevention in individuals with neurological disorders or the elderly. Incorporating multidirectional fall simulations in line with modified constraint-induced movement therapy, the device's efficacy was evaluated by measuring the distance traveled and peak acceleration under different static loads (20, 30, and 40 kg) and input accelerations (1, 2, and 3 m/s^2^). A pilot study with 10 subjects was conducted to assess device performance, utilizing repeated measures analysis of variance and Bonferroni's post hoc analysis. Results indicated a load-dependent reduction in distance traveled, with an average mean difference of 0.74–1.23 cm between the 20 and 40 kg loads for trials of 9 and 18 cm, respectively. Despite varying loads, the device consistently achieved near-anticipated peak accelerations, suggesting its capability to induce effective perturbations. The study also observed a significant lateral movement preference, suggesting adjustments to pulse width modulation and time period may optimize lateral movement performance.

## 1. Introduction

Perturbation-based balance training (PBT) is a promising approach for improving balance control in individuals who have experienced a loss of balance due to aging [1] or neurological conditions [2, 3]. Depending on the physical condition of a person, recommendations are made by medical practitioners to undergo stance perturbation or gait perturbation (perturbation while walking) training. A person who can hardly walk is recommended to initiate stance perturbation training.  Table 1 presents various stance perturbation techniques/technologies that have been shown to effectively enhance the health status of individuals experiencing balance issues. Adjusting perturbation direction and intensity is vital for enhancing the efficacy of balance training devices, as these factors significantly influence the outcome of perturbation-based training [23–27]. Multidirectional perturbations can prevent anticipatory postural adjustments, fostering genuine compensatory steps [23]. Different fall types, such as forward falls leading to wrist fractures [24] and slip-induced falls causing hip fractures [25, 26], emphasize the importance of varied perturbation training. This unpredictability challenges trainees to adapt to unexpected perturbation directions, improving their ability to prevent falls across different scenarios. As trainees' abilities improve, progressively increasing the intensity of perturbations ensures continued advancement and adaptation, enhancing their overall balance and fall-prevention skills.

Unidirectional PBT mechanisms like the lean and release method [8–14], tether release method [15–17], and rubber sheet method [7] prepare trainees for anticipated falls, leading to postural adjustments before perturbation [28]. However, these methods and devices, like the foam test and biodex [20–22], fall short in effectively training for compensatory stepping, unlike waist pull techniques [4–6] that promote lateral stepping to mimic less common push or pull falls. By pulling subjects to either their left or right side, these techniques simulate a fall and encourage compensatory lateral steppings, such as cross-step-front, cross-step-back, or medial sidestep [29]. In contrast, the Radboud Falls Simulator (RFS) offers an advanced eight-directional perturbation capability [18], yet its large size and cost limit accessibility, illustrating the need for versatile yet practical PBT solutions. Our review highlights limitations in current stance PBT devices, including the lack of quantifiable intensity measures in manual therapist-led push-pull methods and foam techniques. Recognizing this critical gap, we are motivated to explore a novel device design incorporating mecanum wheels to better assess and improve patient progress in balance training.

Mecanum wheels, widely utilized in robotics, industries, and logistics [30], are identified as ideal for a perturbation platform due to their capability for multidirectional movement without orientation change, enhancing portability and allowing precise control over the device's acceleration in all directions. Researchers have used a PBT device that perturbed using the principle of platform movement traveled with a distance of 9 cm intervals with an acceleration that increments with 1 m/s^2^ for the stroke population [18, 19]. The perturbation platform was designed to accommodate a single leg, while the other would act as an active limb to produce a compensatory step. A person who does not anticipate a mediolateral perturbation distributes the body weight equally into the two lower limbs [31].

This training trains the complicated interplay of control required for maintaining a quiet, upright stance and responding to external disturbances, highlighting the complexity of balance management [32, 33]. Therefore, the aim of this study was to design a mecanum-built perturbation-based balance training (M-PBT) device with multidirectional perturbation movement and to analyze its performance with variable loads representing a single-leg weight. In addition, a pilot study was conducted to validate the performance of the M-PBT device with 10 healthy participants. The analysis section of this study will test (1) the influence of load on the distance traveled by the device, (2) the influence of load on the peak acceleration generated by the device, (3) the influence of input acceleration on the peak acceleration generated by the device, and (4) the performance of the M-PBT device in generating perturbations with a dynamic load of human participants. The results of this study are expected to provide significant insights into the design and effectiveness of the M-PBT device.

## 2. Materials and Methods

### 2.1. Mechanical Design and Control Aspects

Type X mecanum wheel arrangement mode [34] was followed in this M-PBT device design. The wheel was not arranged precisely parallel to each other as the 360° no-radius rotation by the PBT device was not demanded by the objectives of this study. This indeed helped to reduce the size of the device to 16 cm breadth.

Figure 1 shows the block diagram of the proposed device. The M-PBT device frame was made of an aluminum sheet of thickness 0.5 cm with a dimension of 32 cm × 16 cm (*L* × *B*). It contained four DC planetary geared servo motor with specification of 250 W, 200 RPM, 18 V, 140 kg cm. The DC servo motor was connected with a mecanum wheel of 10 cm diameter and width of 5 cm. The mecanum wheel had nine rollers of 4.7 cm in length and a diameter of 1.945 cm. The two motors connected with respective motor drive MDD20A enabled bidirectional control. Two DC output power supply of 24 V and 10 A were used to provide power to the overall device. The CA2596 DC–DC buck converter step-down module converted 24–12 V to supply power to the Arduino Mega 2560. The platform was designed to move in eight directions in response to the switch pressed.

The control system was programed to provide provisions to select the acceleration and distance with the help of the parameters displayed on the LCD (128 × 64). The distance and acceleration values were opted for with the help of the enter and exit switches. The controller section was connected to the M-PBT device via a 3 m length flame retardant low smoke cable (0.5 sq mm × 24 Core) (Figure 2(a)). The controller panel was encapsulated within a fabric panel of the dimension 40 cm × 13 cm × 20 cm (*L* × *W* × *H*). A crucial aspect of the M-PBT device's control strategy, involves the adjustment of the pulse width modulation (PWM) of the motor and the duration of wheel rotation. This adjustment is pivotal for controlling the motor's speed, thereby directly influencing the platform's acceleration and distance traveled. Through adjusting the PWM signal, the device was able to finely tune the motor's speed to match the required acceleration. Additionally, the modulation of the duration for which the wheels rotate allows for precise control over the distance the platform moves. This dual mechanism of control, which combines PWM modulation with time adjustments, ensures that the platform can achieve the desired motion parameters with high precision.

The two main parameters validated in this study are the distance traveled by the device and the peak accelerations achieved by it. The distance traveled by the device was analyzed using Kinovea software. The Kinovea software has been validated as “excellent” with an intercorrelation coefficient (ICC) score > 0.9 to measure distance parameters [35]. The device was moved for two different distances of 9 and 18 cm in all eight directions with loads of 20, 30, and 40 kg. These load categories were opted because a single leg placed by a person on this platform will exert half their weight. To ensure precise distance measurement, we utilized the gold standard AutoCAD print on A0, as shown in Figure 3(c). This allowed us to take advantage of the grid option in Kinovea [33]. Hence, any distance within the grid was calculated with negligible error (ICC value > 0.9) [36]. The A0 sheet containing the AutoCAD print was affixed securely onto a horizontal wooden panel that was firmly attached to the floor level. This measure was taken in order to eliminate any potential interference in the movement of the perturbation device on the mecanum wheel that may have been caused by the inclination of the floor. To capture the movement of the perturbation platform in eight directions on the transverse plane, the iPhone camera was mounted on a selfie stick and positioned 90 cm above the wooden panel, as shown in Figure 4. For the experimental video analysis, an Apple iPhone 7 Plus was employed, recording at 120 FPS with a resolution of 1,920 × 1,080 pixels, to facilitate detailed motion capture and subsequent analysis via Kinovea software. The wooden panel on which the device was tested had a length of 120 cm and a breadth of 90 cm. The design in AutoCAD included a square box with a dimension of 81.961 cm. This square box was used as the area of the grid option in Kinovea software. The grid option was positioned effectively to the four corners of the square, which had luminous stickers of size 0.5 cm diameter. These details can be seen in Figures 2(a) and 3(c). The PWM and time settings of the device were set to run a distance of 9 and 18 cm with different accelerations of 1, 2, and 3 m/s^2^ based on the trial-and-error test conducted before the experiment.

The Delsys trigno wireless sensors were used to measure the peak acceleration of the M-PBT device. The Delsys inertial measurement unit (IMU) sensor that contains an accelerometer has a measurement range of ±16 g and a sampling frequency of 148 Hz. The nonlocomotion noises were eliminated with the help of an inbuilt low pass filter of 10 Hz [37] in the LabChart (AD Instruments), where the output was exported to Microsoft Excel. Two IMU (IMU1 and IMU2) sensors were placed on the front side of the platform carefully with double-sided adhesive tape. The placement procedure of the Delsys IMU sensor, as recommended in one research study [38], was followed to reduce low cross-axis sensitivity and zero-g offset caused by the default geometric irregularity present in the Delsys IMU sensor. The IMU1 was placed with an *X*-positive side facing the front side of the platform and *Y*-positive on the left side. The IMU2 had *X*-positive facing the backside and *Y*-positive toward the right side of the platform (Figure 2(b)). IMU sensor axis used for analysis with respect to direction is tabulated in Table 2.

We differentiated the trials based on the acceleration and distance traveled by the platform. We conducted 9 and 18 cm trials with different accelerations of 1, 2, and 3 m/s^2^ for 20, 30, and 40 kg loads. The selection of 3 m/s^2^ as one of our acceleration parameters was informed by existing literature, which has demonstrated that this level is both effective and safe for evoking balance reactions without compromising participant safety [18, 39]. Therefore, a total of 18 trials were conducted for straight-line and another 18 trials for diagonal directions. Straight-line trials had forward, backward, left, and right movement, whereas diagonal trials had left forward, right backward, right forward, and left backward. A straight-line or diagonal trial covered a total of four movements repeated twice. The order of movement recorded was as follows: (for straight-line) forward, backward, backward, forward, right, left, left, and right. For diagonal direction, the order followed was left forward, right backward, right backward, left forward, right forward, left backward, left backward, and right forward. Hence, we received eight readings for each trial in straight-line and eight for diagonal. Kinovea measured (Figures 3(a) and 3(b)) all the 16 values generated for a single acceleration and load value. Hence, a total of 16 × 9 = 144 readings were obtained for each 9 and 18 cm trial. The diagonal directional movement required a higher PWM value than the straight-line; hence, analysis was conducted separately for this fact. A Kinovea marker was fixed at the front central region of the M-PBT device (between the Delsys sensor) as a point of reference for the Kinovea software to track the initial and final location for each directional movement.

### 2.2. Participant Description and Pilot Study Experimental Setup

Ten healthy participants were recruited for the pilot study, all of whom had no known issues with balance or mobility. The group comprised of two female and eight male participants, with a mean age of 27.2 ± 5.8 years, a mean height of 167.9 ± 10.2 cm, and a mean weight of 66 ± 9.7 kg. Prior to the study, all participants provided informed consent, and ethical clearance was obtained from the Institutional Ethics Committee of SRM MCH and RC, Tamil Nadu, India.

During the pilot study, it was found that achieving equal weight distribution for the single-leg perturbation was challenging when one leg was placed on the floor and the other on the M-PBT. To address this issue, the nondevice leg was kept on the same level as the device, which was found to be the only feasible option, as shown in Figure 5. The participants wore a fall arrest system to prevent any possible falls that may occur during the pilot study. The key to this fall arrest system lies in the personalized adjustment of the rope's length for each participant. This length is calibrated so that the rope remains slack during normal standing and movement, ensuring no interference with the participant's natural motions or the experimental tasks. If the participant falls to a lower height, which indicates a fall, the rope's length will reach its maximum limit. At this point, the rope will bear the weight of the participant and prevent the fall from continuing. All the participants used their right leg to place on the device, and the left leg was grounded. For this study, a perturbation intensity with an acceleration of 3 m/s^2^ and a distance of 18 cm was set on the device. Apart from this modification, all other experimental procedures were the same as in the validation study.

### 2.3. Statistical Analysis

In order to ensure the performance of the device to produce distance and peak acceleration regardless of the load on the device, it is important to provide consistent output for all loads. To achieve this, we conducted both univariate and multiple comparison tests to determine if there were any variations in performance when producing similar distance and peak acceleration for different loads. The univariate test was conducted to validate the distance and peak acceleration produced by the M-PBT device. Multiple comparisons using Tukey's post hoc analysis were conducted to check the interaction between distance with respect to different load effects and the interaction of peak acceleration with respect to different load effects. The same analysis was also made to find the interaction between peak acceleration with different acceleration inputs provided to the M-PBT device. For the pilot study, a repeated measures analysis of variance (ANOVA) was conducted to test whether, within participants, the distance and acceleration performance of the M-PBT worked equally as they applied dynamic load on the device. It was followed by a pairwise comparison using Bonferroni's post hoc to analyze whether, within each direction of the device, peak acceleration and distance performance were significantly the same or different.

## 3. Results

The data in Table 3 show that the M-PBT device consistently reached the set distance targets during the trial. The overall performance of the distance traveled by the device when applying an input to generate 9 and 18 cm in straight-line and diagonal directions shows reasonable results close to the expected distance (refer to Table 3).

The result section is divided into three sections according to the study objective.

### 3.1. Influence of Load on Distance Traveled by the Device

The distance traveled by the device was 9 and 18 cm with three loads. The result was expected to be statistically nonsignificant to prove that all different loads produced the same distance. The study was statistically nonsignificant for 9 cm straight-line trials with lower load values. The remaining trials in diagonal and higher loads were statistically significant, suggesting that the higher the load, the distances traveled by the M-PBT device were not the same (Table 3). The result also suggests that the distance traveled by the M-PBT device got shorter when the load was increased.

### 3.2. Influence of Load on the Peak Acceleration Generated by the Device

The interaction of the peak acceleration (Delsys) produced with different loads for each input acceleration was analyzed (Table 4). The result shows that all the mean differences between peak acceleration with different loads in the analysis were nonsignificant. It suggests that there is no difference between the peak acceleration generated with different loads. To reiterate, the influence of the load was not evident from the peak acceleration generated by the perturbation device.

### 3.3. Influence of Input Acceleration on the Peak Acceleration Generated by the Device

The output peak acceleration was analyzed by comparing the peak accelerations generated at different input accelerations to the M-PBT device. The study was statistically significant (Table 5). It suggests that all the peak accelerations generated by the device were different from one another.

### 3.4. Influence of Input Acceleration on the Peak Acceleration Generated by the Device

The output peak acceleration was analyzed by comparing the peak accelerations generated at different input accelerations to the M-PBT device. The study was statistically significant (Table 5). It suggests that all the peak accelerations generated by the device were different from one another.

### 3.5. Influence of Dynamic Load Applied by the Participants on Distance Traveled and Peak Acceleration by the Device

In the pilot study, a repeated measures ANOVA was conducted to compare the performance of peak acceleration and distance traveled by the device between participants. The analysis showed a nonsignificant result for peak acceleration (*p*=0.523) and a marginally nonsignificant result for distance traveled (*p*=0.135).

Post hoc tests were conducted to examine the differences in distance and peak acceleration values generated during the movement of the device in eight different directions. Based on the post hoc analysis, it was evident that the directions “right” and “forward right” had a significantly higher peak acceleration compared to other directions within the device (as shown in Figure 6). In terms of distance covered, the directions of “right,” “forward right,” and “backward right” showed significant differences compared to the other directions, as depicted in Figure 7.

## 4. Discussion

The purpose of this research was to design a device named M-PBT and evaluate its effectiveness by subjecting it to multidirectional perturbation movements under different load conditions. We aimed to measure the device's performance by recording the distance traveled and peak acceleration in response to varying loads and input accelerations. Furthermore, we conducted an exploratory pilot study involving ten healthy participants to gain preliminary insights into the device's potential for facilitating balance training. This initial assessment focused on exploring the device's capability to generate suitable perturbations for balance improvement rather than providing conclusive validation of its effectiveness.

The main challenge while designing a PBT device is to replicate a natural fall setting, especially when it has to simulate the exact slip or a trip scenario. In a research study [27], a split treadmill was used to simulate a trip. One belt was set to move faster to accommodate one leg, while the other belt ran at a normal speed. The same study simulated slip by running one belt slower compared to other belts with a comfortable speed. We followed the study [40] that executed slip with the principle of a treadmill belt that moves forward with a reasonable acceleration to result in a backward fall and trip with a treadmill belt backward movement to result in a forward fall. However, in this study, the treadmill has been replaced with an M-PBT device for PBT that is locomoted in multiple directions to simulate slip and trip scenarios.

The mecanum wheel platform enables seamless directional movement while maintaining its orientation. This feature ensures that the leg of a person placed on the platform remains do not get twisted. The device promises multidirectional movement, but the study primarily focused on testing the effects of variable load interactions with peak acceleration and distance the device produced.

### 4.1. Influence of Load on Distance Traveled by the Device

The study shows that the load influences the distance the M-PBT device traveled. The average mean difference between the 20 and 40 kg load for 9 and 18 cm was 0.74 and 1.23 cm, respectively. The result (Table 3) indicates that an increase in the load influenced the M-PBT device to reduce the distance to approximately 1 cm. The mecanum wheel consists of nine rollers made up of rubber material. At a given moment, the small rolling area of the roller touches the ground, which generates enough friction to locomote the device [41]. However, as the load was increased to 40 kg, the rollers tend to deform. The deformation of the roller resulted in an increased surface area at the point of contact with the ground [42]. This may have increased friction and could have reduced the distance traveled by the device.

By increasing either the input PWM or the rotational time period of the motor, the shortage in the distance due to increased load can be corrected. The increase in PWM proportionally increases the peak acceleration and, thereby, the distance of the device; hence, it is crucial to analyze the input PWM and time period fed to the device.

### 4.2. Influence of Load on the Peak Acceleration Generated by the Device

The expectation was that the M-PBT device would generate a corresponding peak acceleration for input acceleration of 1, 2, or 3 m/s^2^, even when loaded with different weights. The findings, as presented in Table 4, corroborated with the expectation suggesting that the interaction of peak acceleration (measured by Delsys) produced with different loads was nonsignificant. Furthermore, the result also suggests that peak acceleration was not reduced by the M-PBT device, which resulted in a shortage of distance when loads were increased. At this point, a deformed roller due to heavier loads was believed to be the reason for the reduced distance the device traveled, and the expectation was to have a reduced peak acceleration. Since there was no effect of load on the M-PBT device to reach peak acceleration, it is suggested that the reason for the reduced distance explained in the first objective may be due to the slippage of the roller that is reported to occur in mecanum mobile robots [43]. Although the distance traveled by the M-PBT device was affected, peak acceleration during its travel was picked up by the M-PBT device.

### 4.3. Influence of Input Acceleration on the Peak Acceleration Generated by the Device

For each trial with varying distance and direction, the motor was supplied with a range of input parameters such as time period and PWM, as listed in Table 5. Additionally, from the above-explained objective, it was inferred that the peak accelerations generated are not impacted by the load. Hence, it was crucial to examine whether the projected peak acceleration input led to the real peak acceleration produced by the M-PBT device during various distance trials. The result shows that the mean peak accelerations were close to the anticipated input value. Moreover, the interaction of these peak accelerations while the device was operated at different distances and motion directions suggested that all the peak accelerations generated were not overlapping, and the differences reflected in Table 5 are significant.

In this study, the M-PBT device was targeted to accommodate a single leg placed at a height of 10 cm. Even though the objective of single-leg perturbation was to reduce the size to make it a portable device, it possesses the principle of modified-constraint-induced movement therapy (mCIMT). M-PBT device was designed to regain balance for a person with a neurological disorder, who lacks the motivation to use the weak leg, especially the individual with a hemiparetic condition. CIMT mainly restricts completely an effective limb (usually used in the upper limb), so the weaker limb was mandated to be used to execute any given task [44]. The lower limb cannot be imposed a complete restriction as humans are bipedal in nature, and two legs are vital in almost all tasks. Thus, the partial restrictions applied to the lower limb make it a type of mCIMT device. The M-PBT device induces perturbation on a single leg, disturbing the center of mass, which makes the other limb to be utilized to realign the center of mass back to the base of support to regain balance. However, the claimed mCIMT property of this device needs real-time study with older people and people with neurological disorders.

### 4.4. Influence of Dynamic Load Applied by the Participants on Distance Traveled and Peak Acceleration by the Device

The performance of the M-PBT device may cause the platform to move a bit more distance and accelerate quickly during lateral movement. In both cases of peak acceleration (shown in Figure 6) and distance traveled (shown in Figure 7), the platform moved significantly more towards the right side for participants using their right leg on the platform. This may be due to the participants feeling more comfortable with the wider stance, which provides them with an increased base of support and stability. This finding is consistent with previous research that has shown that a wider base of support can improve balance and stability [45]. Additionally, nonathletic normal subjects tend to exert greater muscle torque with their hip abductor muscles compared to their hip adductor muscles, which could contribute to this effect [46]. The higher torque of the abductor muscles may assist with the platform movement during lateral movement. It is conceivable that the study participants were able to effectively transfer their body weight while laterally moving their legs, potentially contributing to the movement of the platform in that direction. However, it is important to note that body weight does not aid in the medial direction movement of the platform, as it does in lateral movement (Figure 7). These findings offer valuable insights into the functionality of the M-PBT device during both lateral and medial movements, highlighting the crucial role that body weight and muscle torque play in device performance.

The pilot study involving only ten healthy participants has produced preliminary findings about the M-PBT device's functionality during balance tasks. Results suggest that adjustments to the PWM and time period could enhance the device's performance during lateral movements. However, caution should be exercised in interpreting the results due to the small sample size. A larger and more diverse participant cohort is required to validate the observed trends and comprehensively assess the device's efficacy for individuals with balance issues. Therefore, while the pilot study provides useful directions for future research, further studies are necessary to fully explore the potential benefits of the M-PBT device for balance training.

### 4.5. Limitations and Future Works

In our research, we utilized a wooden panel and an A0 sheet as the surface for the M-PBT device to move on. However, it would be practical to test the device with a wider range of flooring materials that are commonly found in a patient's living environment, such as tiles, marble, or cement. This will necessitate adjusting the input settings based on the floor material, ensuring precise distance and acceleration readings. We also observed a slight deviation in movement angle when using the M-PBT device (as shown in Figures 3(a) and 3(b)). Further investigation is needed to fully understand the impact of this deviation on individuals during straight-line and diagonal movements. Test–retest studies are required to assess the accuracy of the M-PBT device in measuring angle deviation.

## 5. Conclusion

This study suggests that the mecanum wheels can be used for PBT due to their portability, ability to simulate multidirectional falls, and compatibility with mCIMT principles. However, to fully establish their reliability for PBT, further research is necessary. Future studies should focus on overcoming challenges such as slippage and load-bearing limitations to enhance system reliability. Addressing these areas is crucial for advancing the PBT system's effectiveness and safety, promising a significant impact on therapeutic interventions for balance improvement. By prioritizing these research directions, we can move closer to optimizing the PBT system to meet the diverse needs of individuals requiring balance training.

## Figures and Tables

**Figure 1:** Block diagram of the mecanum-built PBT device.

**Figure 2:** (a) Device on the printed sheet on the leveled base and (b) sensor alignment and movement direction.

**Figure 3:** (a) Straight-line measurement (Kinovea output), (b) diagonal measurement (Kinovea output), and (c) AutoCAD design.

**Figure 4:** Experimental setup.

**Figure 5:** Pilot study setup.

**Figure 6:** Pairwise comparison of acceleration generated across various directions by the device when operated at the input acceleration of 3 m/s^2^: results from the pilot study. The  ^*∗*^ and ^#^ have *p*-values less than 0.001 and 0.025, respectively.

**Figure 7:** Pairwise comparison of distance traveled across various directions by the device with expected input distance of 18 cm: results from the pilot study. The  ^*∗*^ has a *p*-value less than 0.001.

**Table 1:** State-of-the-art perturbation training techniques.

Perturbation technology/system	Perturbating principle	Direction of perturbation	Anticipatory strategy	Portability	Parameter reproducibility	Resultant of perturbation action	Cited articles
Motorized waist pulls	Lateral fall perturbation	Bi	Yes	Yes	Yes	Compensatory stepping	Borrelli et al. [4], Yungher et al. [5], Young et al. [6]
Rubber sheet with motor	Platform beneath pulled	Uni	No	Yes	Yes	Compensatory stepping	Weerdesteyn et al.[7]
Lean and release	Cable release	Uni	No	Yes	Yes	Compensatory stepping	Schinkel-Ivy et al. [8], Mansfield et al. [9], Chan et al. [10], Inness et al. [11], Rydalch et al. [12], Inness et al. [13], Lakhani et al. [14]
Tether release	Cable release	Uni	No	Yes	Yes	Compensatory stepping	Van Liew et al. [15], Legg et al. [16], Cortes et al. [17]
Radboud falls simulator	Motorized platform	Multi	Yes	No	Yes	Compensatory stepping	Schinkel-Ivy et al. [18], de Kam et al. [19]
Foam	Foam density	Multi	No	Yes	No	Adjusting weight-bearing joints	Huang et al. [20]
Biodex	Platform inclines	Multi	Yes	No	Yes	Adjusting weight-bearing joints	Gusi et al. [21], Nel et al. [22]

**Table 2:** Delsys connection and the values taken for analysis (refer Figure 2(b)).

Direction	IMU1				IMU2				Peak acceleration
	*X*+	*X*−	*Y*+	*Y*−	*X*+	*X*−	*Y*+	*Y*−	Values taken from sensor axis
Front	√	—	—	—	—	—	—	—	IMU1 *X*+
Back	—	—	—	—	√	—	—	—	IMU2 *X*−
Left	—	—	√	—	—	—	—	—	IMU1 *Y*+
Right	—	—	—	—	—	—	√	—	IMU2 *Y*+
Forward left	√	—	√	—	—	—	—	—	$\sqrt{{\left(IMU1X+\right)}^{2}+{\left(IMU1Y+\right)}^{2}}$
Backward right	—	—	—	—	√	—	√	—	$\sqrt{{\left(IMU2X+\right)}^{2}+{\left(IMU2Y+\right)}^{2}}$
Forward right	√	—	—	√	—	—	—	—	$\sqrt{{\left(IMU1X+\right)}^{2}+{\left(IMU1Y-\right)}^{2}}$
Backward center	—	—	—	—	√	—	—	√	$\sqrt{{\left(IMU2X+\right)}^{2}+{\left(IMU2Y-\right)}^{2}}$

**Table 3:** Examining interaction via multiple comparisons: a comparison of distance generated by various weights.

Load (kg)	Mean difference in distance (*p*-value)				
	20	30	40	Task	Mean distance (cm)
20	—	**0.259 (0.514)**	0.732 (0.007)	9 cm straight	8.906
30	**−0.259 (0.514)**	—	**0.473 (0.116)**		
40	−0.732 (0.007)	**−0.473 (0.116)**	—		

20	—	0.774 (0.000)	1.254 (0.000)	9 cm diagonal	9.260
30	−0.775 (0.000)	—	0.479 (0.014)		
40	−1.25 (0.000)	−0.479 (0.014)	—		

20	—	0.895 (0.008)	1.702 (0.000)	18 cm straight	17.657
30	−0.895 (0.008)	—	0.807 (0.018)		
40	−1.702 (0.000)	−0.807 (0.018)	—		

20	—	**0.341 (0.688)**	1.380 (0.004)	18 cm diagonal	17.875
30	**−0.341 (0.688)**	—	1.038 (0.038)		
40	−1.380 (0.004)	−1.038 (0.038)	—		

The bold values indicate the statistically nonsignificant data, with a *p*-value > 0.5.

**Table 4:** Multiple comparisons of peak acceleration for various applied loads.

Loads (kg)	Mean acceleration difference in m/s^2^ (*p*-value)			Input acceleration (m/s^2^)
	20	30	40	
20	—	0.0362 (0.865)	0.1306 (0.159)	1
30	−0.0362 (0.865)	—	0.0945 (0.378)	
40	−0.1306 (0.159)	−0.0945 (0.378)	—	

20	—	0.1059 (0.848)	0.2563 (0.385)	2
30	−0.1059 (0.848)	—	0.1504 (0.718)	
40	−0.2563 (0.385)	−0.1504 (0.718)	—	

20	—	0.2079 (0.577)	0.1222 (0.826)	3
30	−0.2079 (.577)	—	−0.0857 (0.910)	
40	−0.1222 (0.826)	0.0857 (0.910)	—	

**Table 5:** Peak-acceleration analysis.

Time	PWM			Mean acceleration difference in m/s^2^ (*p*-value)			Task
		Acceleration		1	2	3	
		Input	Actual mean				
7	33	1	1.26	—	−0.814 (0.000)	−1.551(0.000)	9 cm straight
4	50	2	2.08	0.814 (0.000)	—	−0.737 (0.000)	
3	60	3	2.82	1.551 (0.000)	0.737 (0.000)	—	

10	33	1	0.94	—	−1.026 (0.000)	−1.967 (0.000)	9 cm diagonal
4	60	2	1.96	1.026 (0.000)	—	−0.941 (0.000)	
3	83	3	2.91	1.967 (0.000)	0.941 (0.000)	—	

9	43	1	1.06	—	−1.296 (0.000)	−1.888 (0.000)	18 cm straight
6	63	2	2.19	1.296 (0.000)	—	−0.592 (0.013)	
4	102	3	2.95	1.888 (0.000)	0.592 (0.013)	—	

17	33	1	0.87	—	−1.462 (0.000)	−2.048 (0.000)	18 cm diagonal
4	120	2	2.32	1.462 (0.000)	—	−0.586 (0.010)	
3	150	3	2.92	2.048 (0.000)	0.586 (0.010)	—	

## Data Availability

The data that support the findings of this study are available upon request. We are committed to making our data accessible and reproducible, and we encourage interested researchers to contact us for more information.
